# An Improved Transition Probability Matrix for Crime Distribution Prediction

**DOI:** 10.1155/2022/3925503

**Published:** 2022-08-10

**Authors:** Junhao Zhang, Kaicun Zhang, Weiping Li

**Affiliations:** ^1^Department of Image and Network Investigation, Railway Police College, Zhengzhou 450003, China; ^2^Department of Public Security Basic Education and Research, Railway Police College, Zhengzhou 450003, China

## Abstract

The occurrence of crime has always been the main problem affecting urban public security and social security environment. Therefore, the prevention and control of crime is the focus of public security work. The traditional police strategy has poor timeliness and cannot respond and adjust in real time with the occurrence of criminal activities, and its deterrence and control of criminal activities are limited. To address the problem of low accuracy of existing crime distribution prediction models, an improved transition probability matrix for crime distribution prediction is proposed in this paper. Based on a large number of trajectory data of criminals, this paper quantitatively describes the temporal and spatial characteristics of crowd movement in different areas of the city by using the temporal and spatial transfer probability. Then, combining Markov chain and Bayes' theorem, the probability model of spatio-temporal transfer of criminal groups in regions is constructed. Finally, the model predicts the number of crimes in urban grid areas.

## 1. Introduction

Crime is a social problem that cannot be ignored in the process of urban development [1]. With the development of science and technology and the concentration of social wealth, the phenomenon of crime is more frequent, intelligent, and destructive. The analysis of the current situation of criminal behavior and the prediction of criminal trend can restrain the growth of crime rate, effectively promote the public security organs to strengthen the law enforcement, and maintain social stability [2]. At present, crime prediction has become an important work for the public security organs to prevent and crack down on crimes, which plays an increasingly significant supporting role in police work [3]. With the development of big data sampling and Internet information processing technology, more and more attention has been paid to the correlation between criminal behavior and social factors, economic factors, and environmental factors in the studied area [4].

The purpose of crime spatio-temporal analysis is to predict the time, place, and type of crime according to the historical crime data [5]. Its research is of great significance to the maintenance of public security and attracts more and more attention in academic circles. Researchers often use a number of classic machine learning and pattern recognition methods to solve this problem. However, previous studies have neglected the full combination of historical crime data and socio-environmental factors [6]. Previous studies on spatio-temporal analysis of crime are usually based on historical crime data. Classical machine learning and pattern recognition methods are used to model and predict this problem, including linear regression algorithm, auto regression algorithm, lasso regression algorithm, ridge regression algorithm, decision tree algorithm, and Bayesian algorithm [7–11].

Other studies focus on how to introduce machine learning algorithms into spatio-temporal models to obtain a series of spatio-temporal results on crime problems. Literature [12] introduced a regressive integral moving average (ARIMA) model to study the crime rate prediction of a city in a few weeks. By comparing existing studies, it can be seen that in terms of spatio-temporal analysis of crimes, Apriori algorithm is based on the principle of support, confidence, and promotion criteria to screen out strong association rules [13]. When attribute data is too much or the amount of data is too large, it is difficult to mine association rules with predictive significance because of low support. Random forest, LightGBM, and other decision tree algorithms have better effect on category analysis of criminal events [14]. However, the temporal and spatial connection of the crime is vague and cannot be described concretely.

The current research on regional population prediction is generally extended from individual prediction to population prediction. However, due to the large population in urban areas, the calculation amount is too large. Moreover, the impact of the uncertainty of individual prediction on population prediction at the urban regional scale also needs to be further studied, and an efficient prediction method at the population level needs to be established [15]. Studies on time series prediction mainly focus on the temporal variation of regional population, but seldom consider the dynamic cumulative impact of population movement in reality [16]. The predictors based on Markov model take into account the number of people in the region and the characteristics of crowd transfer in the current period as the prediction law of the next period [17]. However, the accuracy of the prediction will be affected due to the spatial and temporal differences in human motion.

Therefore, this paper adopts crime location data from a group perspective. Considering the spatio-temporal difference of crowd movement, a prediction method for the number of criminals on the urban regional scale is proposed, which combines Markov chain and Bayes' theorem. The method calculates the probability of spatio-temporal shift of crime location and constructs the prediction model of crime number to predict the crime number in urban area.

The innovations and contributions of this paper are as follows:

1. The algorithm model in this paper makes full use of the historical track data of criminals to describe the space-time characteristics of crowd flow in different regions
2. Fully combining the advantages of Markov chain and Bayes' theorem, to form a partition prediction model.
3. The distance factor is added into the model, and the change of movement law in adjacent periods is considered

This paper consists of four main parts: the first part is the introduction, the second part is methodology, the third part is result analysis and discussion, and the fourth part is the conclusion.

## 2. Methodology

### 2.1. Space-Time Transfer Probability

Transition probability is an important concept in Markov correlation theory. It is used to describe the transition process from one state to the next in the state space. According to the definition of Markov theory, the transition probability of state *t* Markov chain {*I*_*t*_, *t* ∈ *N*} is set as conditional probability  *u*_*i*_*t*_,*i*_*t*+1__^*t*^, and the calculation formula is shown in the following equation:

(1) $$\begin{array}{c} u_{i_{t},i_{t+1}}^{t}=U\left\{I_{t+1}=i_{t+1}\;|\;I_{t}=i_{t}\right\}, \end{array}$$

where *u*_*i*_*t*_,*i*_*t*+1__^*t*^ represents the probability of the state changing from *i*_*t*_ to *i*_*t*+1_ from the current state *t* to the next state *t*+1.

The spatial position of the criminal at time *n* is expressed as *X*_*t*_=(*longitude*_*t*_, *latitude*_*t*_, *n*), where *n* represents the time. (*longitude*_*t*_, *latitude*_*t*_, *n*) indicates the longitude and latitude coordinates of the administrative area where the offender is located, abbreviated as (lo*n*_*t*_, *lat*_*t*_). The spatial position of criminals at different time constitutes the moving trajectory *L*_*t*_=(*X*_0_, *X*_1_, *X*_2_,…, *X*_*t*_), where *t* is the number of track records. In this paper, the change of spatial position is regarded as the change of state. *X*_*t*_=(*lon*_*t*_, *lat*_*t*_, *n*) as the state  *i*_*t*_. Corresponding state of underground *i*_*t*+1_ is expressed as *X*_*t*_=(*lon*_*t*+1_, *lat*_*t*+1_，*n*+1). Transition probability of time and space for the location of crime personnel is expressed as *u*_*i*_*t*_*i*_*t*+1__^*n*^=*U*(*X*_*t*+1_∣*X*_*t*_).

The spatio-temporal transfer probability of criminals' location is used to quantitatively describe the possibility of criminals moving between different regions. From the location data of active region, the number of criminals in each region can be counted  *T*_*x*_^*n*^ and *flow*_*x*,*y*_ represents the number of criminals between region *x* and region  *y* and *flow*_*x*,*y* _^*n*^ represents the number of times that the current location is *x* and the next location is *y* in the trajectory of criminals in time period *n*. According to Bayes' theorem, the space-time transfer probability *u*_*x*,*y*_^*n*^ of criminals from region *x* to region *y* is calculated by the following formula:

(2) $$\begin{array}{c} u_{x,y}^{n}=u\left(X_{y}|X_{x}\right)\\ =\frac{u\left(X_{y}\right)u\left(X_{x}|X_{y}\right)}{\sum_{z=1}^{w}u\left(X_{z}\right)u\left(X_{x}|X_{z}\right)}\\ =\frac{\left(T_{y}^{n+1}/T^{n+1}\right)\left({\text{flow}}_{x,y}^{n}/T_{y}^{n+1}\right)}{\sum_{z=1}^{w}\left(T_{z}^{n+1}/T^{n+1}\right)\left({\text{flow}}_{x,z}^{n}/T_{z}^{n+1}\right)}\\ =\frac{{\text{flow}}_{x,y}^{n}}{\sum_{z=1}^{w}{\text{flow}}_{x,z}^{n}}. \end{array}$$

Here, *x* and *y* represent the area where the criminal is located in time period *n* and time period *n*+1, respectively, *w* represents the number of criminals in the administrative region, flow_*x*,*y*_^*n*^ represents the number of criminals moving from region *x* to region *y* in time period *n*, *T*_*y*_^*n*+1^ represents the number of criminals in area *y* in time period *n*+1, and *T*^*n*+1^ is the number of criminals in all areas of *n*+1.

### 2.2. Space-Time Transition Probability Matrix

A space-time transition probability matrix can represent the likelihood of a criminal moving between regions.  Figure 1 shows a schematic diagram of inter-regional crowd flow. When only considering the movement of criminals from single region *x* to *w* regions (Figure 1(a)), criminals move from region *x* to region 1,2,…, *w*, temporal and spatial transfer probability form a row vector *U*_*x*_^*n*^, can be expressed as *U*_*x*_^*n*^=[*u*_*i*,1_, *u*_*i*,2_, ⋯, *u*_*i*,*w*_].

Figure 1(b) shows a schematic diagram of criminals moving between multiple areas. The spatial-temporal transfer probability of crowd movement between multiple regions can be expressed as a two-dimensional *w* × *w* matrix *U*^*n*^, as shown in the following equation:

(3) $$\begin{array}{c} U^{n}=\left|u_{xy}^{x}\right|=\left[\begin{array}{ccccc} u_{11:} & u_{12} & \cdots & u_{1y} & u_{1w}\\ u_{21:} & u_{22} & \cdots & \vdots & \vdots \\ \vdots & \vdots & \cdots & \vdots & \vdots \\ u_{x,1.} & \vdots & \cdots & u_{xy} & \vdots \\ u_{w1} & \cdots & \cdots & \cdots & u_{ww} \end{array}\right], \end{array}$$

where the transition probability matrix *U*^*n*^ satisfies the matrix element 0 ≤ *u*_*x*,*y*_^*n*^ < 1, and the sum of all elements in each row is 1.

### 2.3. Criminal Distribution Prediction Model

#### 2.3.1. Castro's Prediction Model

Castro's model uses the nonaftereffect of Markov chain to predict traffic flow in different periods. Markov effect is a hypothetical random process in which the conditional distribution function of the random variable is only related to itself in the state space and has nothing to do with the state at any previous time. The model assumes that the number of vehicles in urban areas remains constant. At different time granularity, the traffic flow of each time period was counted, and the probability matrix *U*^*n*^ of vehicle temporal and spatial transition was calculated. As shown in formula (4), the traffic flow prediction model is constructed. This model is widely used in the short-term prediction of urban traffic flow. By using the idea of state transfer in Markov chain, the number of criminals in each region in the current period *T*^*n*^ and transition probability matrix *U*^*n*^ can be used to predict the number of criminals in each region in the next period. As shown in following formula:

(4) $$\begin{array}{c} N\_{predict}^{n+1}=U^{n}\times T^{n}, \end{array}$$

where *U*^*n*^ is the transition probability matrix of criminals in time period *n*, *U*^*n*^=|*u*_*xy*_^*n*^|, 0 ≤ *u*_*xy*_ ≤ 1, ∀*x*, *y* ≤ *w*, ∑_*y*=1_^*w*^*u*_*xy*_^*n*^=1, and *T*^*n*^ is the number vector of criminals in each region in time period *n*.

#### 2.3.2. Model Improvement

The prediction method of the number of regional criminals in this paper combines Bayes theory and Markov chain without aftereffect. The time and space transfer probability of criminals between regions are calculated. On the basis of the Castro model, the prediction method of the number of criminals in the region is constructed. The improvement of the Castro model is given in detail in the following two aspects:

(1) In reality, due to inter-regional population flow and other phenomena, the total population in the region is constantly changing, which makes the assumption that the total number of criminals in the model remains unchanged and untenable. In view of the fluctuation of the total number of criminals, this paper uses historical track data to determine the correction of the total number of criminals in adjacent periods.
First, the correction term Δ*T*^*n*⟶*n*+1^ of the number of criminals in the adjacent period is calculated. Training data statistics obtain the number of regional criminals in each period. The variation of the number of criminals Δ*T*^day,*n*⟶*n*+1^ in the adjacent time period of each day was calculated, respectively. The day superscript is used to identify different dates. The training data shows the maximum value Δ*T*_max_^*n*⟶*n*+1^ and the minimum value Δ*T*_min_^*n*⟶*n*+1^. The average is divided into *t* state intervals [*g*]_*z*_ and *h*_*z*_. The probability *u*_*z*_ of Δ*T*_*n*⟶*n*+1_^day^ in each interval [*g*]_*z*_ and *h*_*z*_ is calculated. According to the following formula, the weighted average of the mean value of the interval is used to obtain the correction term Δ*T*^*n*⟶*n*+1^. The mean value of the interval is calculated to minimize the influence of the extreme value of the number of changes caused by emergencies on the number of regional criminals  Δ*T*^*n*⟶*n*+1^.
  (5) $$\begin{array}{c} \Delta T^{n⟶n+1}=\sum_{z=1}^{t}u_{z}\times \frac{1}{2}\left(g_{z}+h_{z}\right), \end{array}$$
where *g*_*z*_ = Δ*T*_min_^*n*⟶*n*+1^ + (*z*/*t*)(Δ*T*_max_^*n*⟶*n*+1^ − Δ*T*_min_^*n*⟶*n*+1^), *h*_*z*_ = *g*_*z*_ + (1/*t*)(Δ*T*_max_^*n*⟶*n*+1^ − Δ*T*_min_^*n*⟶*n*+1^), *z* = 0,1, ⋯, *t* − 1.Δ*T*_max_^*n*⟶*n*+1^, A represents the maximum value of changes in the number of criminals in adjacent periods *n* and *n* + 1 in the training dataset, and Δ*T*_min_^*n*⟶*n*+1^ is the minimum.
Similarly, the correction term  Δ*U*^*n*⟶*n*+1^ of the spatio-temporal transition probability matrix of the population in the adjacent period was calculated. The difference of crowd movement rule in different time periods will lead to the change of temporal and spatial transition probability of crowd movement in different regions. The correction term Δ*U*^*n*⟶*n*+1^ of the space-time transition probability matrix reflects the difference in the crowd's movement characteristics in different periods. The calculation is based on Δ*u*_*x*,*y*_^day,*n*⟶*n*+1^, the difference of space-time transfer probability between region *x* and *y* in the matrix. The correction term *u*_*x*,*y*_^*n*^ and *u*_*x*,*y*_^*n*+1^ of the transfer probability is from the transfer of *n* and *n* + 1 in the adjacent period of each. The difference value of transfer probability between region *x* and region *y* is calculated. The difference value of transfer probability Δ*u*_*x*,*y*_^day,*n*⟶*n*+1^ between regions in adjacent time periods of every day is divided into *t* intervals, and the correction term of space-time transfer probability Δ*u*_*x*,*y*_^*n*⟶*n*+1^ between regions *x* and *y* is calculated according to the following equation. We can get from this, the adjacent time and the crowd moving time of transition probability matrix correction item Δ*U*^*n*⟶*n*+1^ = |Δ*u*_*x*,*y*_^*n*⟶*n*+1^|(*x*, *y* = 1,2,…, *w*).*w* is the predicted number of this area.
  (6) $$\begin{array}{c} \Delta u_{xy}^{n⟶n+1}=\sum_{z=1}^{t}u_{z}\times \frac{1}{2}\left(g_{z}+h_{z}\right), \end{array}$$
where
  (7) $$\begin{array}{c} g_{z}=\Delta u_{xy,\min}^{n⟶n+1}+\frac{z}{t}\left(\Delta u_{xy,\max}^{n⟶n+1}-\Delta u_{xy,\min}^{n⟶n+1}\right),\\ h_{z}=g_{z}+\frac{1}{t}\left(\Delta u_{xy,\max}^{n⟶n+1}-\Delta u_{xy,\min}^{n⟶n+1}\right),\\ z=0,1,\cdots ,t, \end{array}$$
where Δ*u*_*xy*,max_^*n*⟶*n*+1^ represents the maximum difference value of spatio-temporal transfer probability between region *x* and region *y* in the training data in adjacent periods and Δ*u*_*xy*,min_^*n*⟶*n*+1^ is the minimum.
(2) Specific to the calculation of changes in the number of crimes in each region. Previously, the flow distribution of Castro's prediction model did not consider the change of the movement law in adjacent periods. In this paper, the correction term Δ*U*^*n*⟶*n*+1^ of the space-time transition probability matrix is added to the model. The improved transition probability matrix *U*^*n*′^ is used to allocate the number of regional criminals Δ*T*^*n*⟶*n*+1^. The actual significance of the correction item Δ*U*^*n*⟶*n*+1^ of the probability of spatio-temporal transfer between regions lies in the quantitative description of the differences in the law of crowd movement between urban regions in different periods of time. According to formula (8), the transition probability matrix *U*^*n*′^ that is closer to the actual user movement rule in time period *n* + 1 can be obtained. I scale *U*^*n*′^ so that it still adds up to 1. Finally, according to the improved transition probability matrix *U*^*n*′^, the change Δ*T*^*n*⟶*n*+1^ of the number of crimes in the interval of *n* + 1 is allocated to each area. According to formula (9), the predicted value of the number of criminals in each region in *n* + 1 period was obtained.
  (8) $$\begin{array}{c} U^{n^{\prime }}=U^{n}+\Delta u^{n⟶n+1}, \end{array}$$
  (9) $$\begin{array}{c} N\_{predict}^{n+1}==T^{n}+\Delta T^{n⟶n+1}\times U^{n^{\prime }}. \end{array}$$

#### 2.3.3. Main Flow of the Algorithm

The basic flow of the algorithm in this paper is shown in Figure 2. The basic process includes three stages: data preparation, model training and model prediction, and evaluation. First of all, the inter-regional flow, *flow*_*x*,*y*_^*n*^, of criminals in different periods of time and the number of criminals in the region *T*^*n*^ are counted. According to formula (2), the spatio-temporal transfer probability of criminal groups in regions is calculated, and the spatio-temporal transition probability matrix *U*^*n*^ is constructed. Then, the historical track data is used to train the prediction model, and the correction terms of the number of criminals in adjacent areas and the transition probability matrix are calculated according to formulas (5) and (6). Finally, formula (9) is used to predict the number of regional crimes. The prediction performance of the proposed algorithm is analyzed and evaluated by the prediction accuracy. The optimal number of training weeks and correction items were determined through experiments.

## 3. Result Analysis and Discussion

### 3.1. Historical Case Analysis and Prediction Experiment Design

#### 3.1.1. Spatio-Temporal Scale and Historical Case Analysis

At present, China's police resources are limited, and the patrol scope of a single police officer is limited. In order to achieve accurate prediction and consider the actual working conditions, the interscale of crime hot spot experimental prediction should not be too large. Therefore, the grid region research method is adopted. According to Griffith et al. calculation formula for grid treatment of the research area, as well as the distribution of actual case point data, the whole research area is divided by 200 m × 200 m grid. Smaller space scales such as 150 m and 50 M are compared. To divide the grid with 200 m × 200 m, the case points will fall into some grids intensively and reduce the contingency of hot spot grids. More stable hot spot grid distribution can reflect the occurrence mechanism and distribution law of cases and improve the accuracy of crime hot spot prediction.

#### 3.1.2. Grid Classification and Prediction Experiment

According to the spatial scale of 200 m × 200 m, the research area was divided into 375 grids. According to the distribution of historical crimes in all biweekly periods from 2017 to 2019, the frequency of cases occurring in each grid was calculated. The optimal number of clusters was determined to be 3 or 4 by *k*-means clustering method. Therefore, all grids are divided into stable hot spot grid, relatively hot spot grid, occasional hot spot grid, and nonhot spot grid. The specific grid distribution diagram is shown in Figure 3. The results showed that there were 20 stable hot spot grids, and the frequency of cases occurred more than 50 times in 78 biweekly grids, and cases occurred in 68 biweekly grids with the highest frequency. There were 36 hot spots with higher incidence, and the frequency of cases occurred was greater than 25 times and less than 44 times in 78 biweekly grids. There were 49 accidental hot spot grids, and the frequency of cases occurred was greater than 15 times and less than 26 times in 78 biweekly periods. In the remaining 270 grids, cases occurred less than 12 times in 78 biweekly periods. There are even parts of the grid that never have a case, so they are classified as nonhot spot grids. The number of grids and cases of each type are shown in Table 1.

After all the grids were classified, improved transition probability matrix prediction models were constructed for the whole study area and all kinds of grids, respectively. The transition probability matrix regards hot spot grid prediction as a dichotomous problem and predicts hot spot grids with cases occurring in the predicted period from all target grids. The number of cases per grid from 2017 to 2019 in the same period as the target period and in 3 adjacent periods were counted. Three representative variables, namely, urban village area, road network density, and POI (catering, shopping mall, and entertainment) density, were selected from the built environment, respectively, as covariables of the crime hot spot prediction model, and the improved prediction model was constructed, and the values of the three built environment covariables corresponding to each grid were calculated. Only historical crime data and two data with historical crime data and three covariables were used as input data. The three algorithms use the same input data as training samples and variables of the data set to be predicted.

### 3.2. Analysis of Prediction Results

#### 3.2.1. Overall Prediction Results of the Study Area

The overall prediction results of the improved transfer matrix model before and after the addition of covariates were compared by two indexes: grid hit ratio *HitR*_*a*_ and case hit ratio *HitR*_*n*_. The calculation formulas of *HitRa* and *HitRn* are shown in formulas (10) and (11), respectively. Based on these two evaluation indicators, the prediction results of 26 biweekly experiments in 2019 are shown in Table 2. The line charts of *HitRa* and *HitRn* of the three model indicators are shown in Figures 4 and 5.

(10) $$\begin{array}{c} HitR_{a}=\frac{a^{*}}{A}, \end{array}$$

where *A* is the total number of actual hot spot grids and *a*^*∗*^ is the number of correctly predicted hot spot grids.

(11) $$\begin{array}{c} HitR_{n}=\frac{n}{N}, \end{array}$$

where *n* is the total number of cases in the research area and *N* is the actual number of cases in the predicted hot spot grid.

According to the average of accuracy evaluation indexes of 26 experimental prediction results, the grid hit ratio (*HitR*_*a*_) and case hit ratio (*HitR*_*n*_) of the prediction results of the improved prediction model in this paper are both higher than those in literature [18, 19], and significant differences are tested at the level of 0.5. In terms of standard deviation, the improved model proposed in this paper has a more stable performance than literature [18] and literature [19] in 26 experiments.

Through the comparative analysis of 2 index line charts, this paper found that in the 26 two-week prediction experiments throughout 2019, the improved prediction model with built environment covariable data has better performance in terms of the overall prediction effect of the study area. Under the same experimental data and requirements, the grid hit ratio and case hit ratio are higher than those predicted by other models. This shows that the model in this paper can correctly predict more hot spot grids. And the hot spot grids correctly predicted have higher crime density and can cover more cases. In this study, the number of hot spots predicted by each biweekly experiment is the same as the actual number of hot spots.

As can be seen from the variation trend of Figures 4 and 5, whether it is literature [18], literature [19], or the prediction model in this paper, the case hit ratio of the prediction experiment results also fluctuates with the rise and fall of the grid hit ratio. In other words, under normal circumstances, the grid hit rate is high and the hit rate of cases in the appropriate period is also high.

#### 3.2.2. Classification Grid Prediction Results

The evaluation index system is optimized before comparing the prediction effect of various grids before and after adding covariates. Since the number of predicted hot spot grids will change after the addition of covariates, a new evaluation index, *HitE*_*n*_, case hit efficiency, is added in addition to the two indexes mentioned above. The calculation formulas of *HitE*_*n*_ is shown in the following formula:

(12) $$\begin{array}{c} HitE_{n}=\frac{HitR_{n}}{a/A}, \end{array}$$

where  *HitR*_*n*_ is the case hit ratio, *a* is to predict the number of hot spot grids and *A* is the actual number of hot spot grids.

Table 3 is a summary of the accuracy of the prediction results of the four types of grids and is the comparison of the results of the stable hot spot grid, relatively hot spot grid, occasional hot spot grid, and nonhot spot grid before and after adding the built environment covariable.

For stable hot spot grid with high incidence, the number of predicted hot spot grid increases, and *HitR*_*a*_ and *HitR*_*n*_ of grid hit ratio are significantly improved after the addition of three covariables. Meanwhile, in terms of *HitE*_*n*_ of case hitting efficiency, the mean value of the improved prediction model proposed in this paper is slightly higher than that in literature [18, 19]. At the same time, it also reflects that the prediction efficiency of the model with the addition of covariables is higher than the original prediction model using only historical crime data, and the actual hot spot grid can be found more “hot.”

For hot spot grids with high incidence, the number of predicted hot spot grids increases, and *HitR*_*a*_ and *HitR*_*n*_ of grid hit ratio are significantly improved after the addition of three covariables. According to *HitR*_*n*_ of case hit efficiency, although the mean value of the improved prediction model proposed in this paper is slightly higher than the results in literature [18] and literature [19], it is not statistically significant. It shows that the overall prediction efficiency is not significantly improved after the addition of covariables. Therefore, the prediction hit ratio can be improved for hot spot grids with high incidence by increasing the number of predicted hot spot grids. The stable hot spot grid and relatively hot spot grid are the areas with high concentration of crimes against property in public places, which need to be taken as the key areas for crime prediction, prevention, and control. As can be seen from the above analysis results, when spatial differentiation is considered, the case hit ratio of the partition model with stable and high hot spot grid can be close to 0.912 and 0.682, respectively. According to the prediction results of the zoning model, more effective monitoring and management can be carried out for these two types of high incidence areas, which is of great significance for crime prediction and prevention in the overall study area. The accuracy of the zonal model is significantly higher than that of the whole model, which also indicates that considering spatial differentiation plays an important role in improving the accuracy of the crime hot spot prediction model. Therefore, it is necessary to establish different zoning models for different types of regions according to the spatial differentiation of crimes. By optimizing the crime hot spot prediction model of each zoning model, the overall prediction accuracy of the study area is improved.

#### 3.2.3. Accuracy of the Prediction Model

In order to check the relationship between the accuracy of the algorithm and the amount of data, an experiment was conducted to add 1000 data as sample data each time. A small amount of data is extracted from the recently acquired data as test data to test the algorithm's accuracy, the algorithm's accuracy under different data amounts is counted, and a broken line graph is drawn. The corresponding results are shown in Figure 6.

According to the analysis in Figure 6, the algorithm's accuracy increases with the increase of sample data. However, when the number of sample data reaches a certain number, the algorithm's accuracy tends to be stable. After 6000 pieces of data, the imported data contains some data that do not conform to objective laws, and it is used as sample data for machine learning. As can be seen from Figure 6, the accuracy of literature [20], literature [21], literature [22] and the prediction model in this paper all declined when the data volume was 7000, but the accuracy still maintained a high level.

#### 3.2.4. Performance Comparison of Prediction Models

In this paper, the distance factor is introduced into the prediction of crime distribution model. In order to better verify the performance of the algorithm presented in this paper, the distance factor was also incorporated into literature [20], literature [21], and literature [22] to predict the distribution of crimes, which was compared with the prediction model presented in this paper. The predicted results are shown in Figure 7. As can be seen from Figure 7, literature [20] performs worst among all the comparison algorithms, especially in regions 1, 2, 8, and 10. From zone 6 to 10, literature [20], literature [21], and literature [22] fluctuated greatly. However, the prediction model proposed in this paper has a relatively mild trend in these areas, and the effect of fitting the actual value is also better than that of other algorithms, showing better performance than that of other algorithms.

## 4. Conclusion

In recent years, with the continuous development of economy and society, the form of comprehensive social governance is increasingly severe. Crimes such as theft and robbery are becoming more and more prominent and can easily induce major social risks. It is very important to construct the prediction model of crime distribution in order to fight against various criminal activities. Based on Markov chain and Bayes' theorem, this paper proposes a method to predict the number of criminals based on the probability of spatio-temporal transition of criminals' location. The prediction method proposed in this paper comprehensively considers the spatio-temporal characteristics of urban population movement and is suitable for regional population prediction at the regional scale of urban grid. The experimental results show that the proposed algorithm quantifies the spatio-temporal characteristics of human movement and has a good prediction accuracy of the number of criminals. However, more experimental studies are still needed to explore the principles and the data used to predict different types of crime in different research areas. In the future, only by further understanding the causes and laws of the occurrence of crime while doing empirical research, we can carry out more effective crime prevention and control, stabilize social security environment, and maintain urban public security through practical measures.

## Figures and Tables

**Figure 1:** Schematic diagram of regional crowd movement. (a) Movement of people in one area. (b) Multiple sections of people moving.

**Figure 2:** Basic procedures of the prediction method.

**Figure 3:** Grid classification by historical crime events in the study area.

**Figure 4:** Prediction results of crime hot spots in the study area in 2019 (grid hit ratio).

**Figure 5:** Prediction results of crime hot spots in the study area in 2019 (case hit rate).

**Figure 6:** Accuracy of each prediction model.

**Figure 7:** Prediction of model performance.

**Table 1:** Number of classified grid cases in the study area during 2017–2020.

Category	Stabilize the hot spot grid	Higher hot spot grid	Occasional hot spot grid	Nonhot spot grid
Total number of networks/unit	25	36	49	270
Actual hot spot grid average/unit	12	16	13	24
Average number of cases/case	16.349	19.578	17.088	25
Number of cases standard deviation/case	5.413	5.149	6.102	7.057

**Table 2:** Prediction results of crime hot spots in the study area in 2019.

	Grid hit ratio *HitR*_*a*_			Case hit rate *HitR*_*n*_		
	Literature [18]	Literature [19]	Proposed	Literature [18]	Literature [19]	Proposed
The average	0.455	0.467	0.479	0.504	0.526	0.534
The standard deviation	0.076	0.072	0.068	0.085	0.083	0.079

**Table 3:** Results of crime hot spot prediction experiment of four kinds of grids in 2019.

	Grid hit ratio *HitR*_*a*_			Case hit rate *HitR*_*n*_			Case hit efficiency *HitE*_*n*_		
	Literature [18]	Literature [19]	Proposed	Literature [18]	Literature [19]	Proposed	Literature [18]	Literature [19]	Proposed
Stabilize the hot spot grid	0.825	0.891	0.914	0.841	0.898	0.912	0.585	0.592	0.597
Higher hot spot grid	0.605	0.631	0.637	0.631	0.679	0.682	0.471	0.474	0.479
Occasional hot spot grid	0.361	0.334	0.376	0.391	0.374	0.418	0.432	0.425	0.436
Nonhot spot grid	0.181	0.175	0.186	0.232	0.225	0.244	0.415	0.491	0.511

## Data Availability

The labeled dataset used to support the findings of this study is available from the corresponding author upon request.
